This article has been retracted.

# FAM87A as a Competing Endogenous RNA of miR-424-5p Suppresses Glioma Progression by Regulating PPM1H

**DOI:** 10.1155/2021/7952922

**Published:** 2021-10-18

**Authors:** Hua Xu, Haiping Zhang, Lina Tan, Yang Yang, Haiyun Wang, Qin Zhao, Jun Lu

**Affiliations:** ^1^Radiotherapy Center, Xi'an International Medical Center Hospital, Xi'an, Shaanxi Province, China 710100; ^2^Department of Geriatric Endocrinology, The First Affiliated Hospital of Xi'an Jiaotong University, Xi'an, Shaanxi Province, China 710100

## Abstract

Far less has been unveiled about the functions of lncRNAs on cancers yet. Here, we reported that lncRNA FAM87A, as a ceRNA of miR-424-5p, played a vital role in glioma development. qRT-PCR result indicated that FAM87A was abnormally downregulated in glioma tissue and cells. Survival analysis suggested that the FAM87A expression was negatively correlated with the survival rate. Effects of FAM87A on human glioma cell lines were also analyzed by MTT, Edu, and transwell assays. FAM87A hastened proliferation and migration of glioma cells. MiR-424-5p, predicted target of FAM87A, was fostered in glioma, which was examined by qRT-PCR. A negative correlation was indicated between FAM87A and miR-424-5p. Results of bioinformatics, dual luciferase, and RIP assays unveiled that FAM87A and miR-424-5p act upon each other. In addition, miR-424-5p targeted 3′-UTR of PPM1H. Also, effects of miR-424-5p/FAM87A on glioma cells were identified via the cell function experiments. FAM87A suppressed PPM1H by binding to miR-424-5p competitively, thereby restraining cell proliferation, migration, and invasion. Collectively, these findings illuminated a new mechanism for glioma progression. Therefore, FAM87A may act as a feasible target for glioma treatment.

## 1. Introduction

Glioma comprises approximately 80% of primary malignant brain tumors [1]. In recent years, surgical resection combining temozolomide (TMZ) chemotherapy is generally used for the treatment of glioma [2]. However, due to strong cell proliferation and invasion capacities of glioma, the therapeutic effect is unfavorable [3]. It is urgent to reveal detailed molecular mechanism of malignant processes of glioma to find out novel therapeutic targets.

Human genome sequence data show that only a small part of total DNA sequence can encode proteins. Hence, most transcripts are noncoding RNAs (ncRNAs) [4]. MicroRNAs (miRNAs), as a family of small ncRNAs, have been extensively studied, especially concerning their functions in the gene expression and cancer-related biological functions [5]. A recent study showed that long noncoding RNAs (lncRNAs) play vital parts in multiple cancers [6]. Some lncRNAs can simultaneously serve as an oncogene, tumor suppressor gene, or both in different environments [7]. Many lncRNAs play a paramount part in the progression of glioma. Chen et al. [8] found that LINC01198 in glioma enhances cell proliferation while inhibiting TMZ resistance by inhibiting the PTEN expression in the NEDD4-1-dependent mode. Jun et al. [9] found that lncRNA TUG1 constrains tumor development by fostering glioma cell apoptosis. LncRNAs are not only directly involved in the biological processes of tumors but also modulate downstream target genes via competitively binding to miRNAs to achieve the regulation of oncogenesis. He et al. [10] reported that lncRNA UCA1 modulates iASPP by competitively binding to miR-182, thereby regulating the proliferation and metastasis of gliomas. However, many lncRNAs have not been studied yet, and their functions in glioma remain unclear.

LncRNA FAM87A has not been fully studied. However, in the study of tumor markers, Zhang et al. [11] found that the ceRNA network based on several hub genes including FAM87A can be applied to predict prognosis status of tongue squamous cell carcinoma patients. Nevertheless, underlying mechanism of FAM87A in glioma progression has not been fully studied.

In our study, FAM87A expressions in glioma tissue and cell lines were detected. Effects of FAM87A on glioma cell behaviors were assessed. Moreover, bioinformatic tools were applied to predict potential miRNA targets which may interact with FAM87A to regulate glioma cell progression. At the same time, downstream target gene (PPM1H) of miR-424-5p was determined. In brief, we reported the FAM87A/miR-424-5p axis, which regulated glioma cell behaviors by targeting PPM1H. Our findings offer novel insights into functions of FAM87A and miR-424-5p in glioma metastasis.

## 2. Materials and Methods

### 2.1. Microarray Analysis

RNA expression and clinical data on glioma were accessed from The Cancer Genome Atlas (TCGA) database. Then, edge*R* was employed for differential expression analysis (∣logFC | >2, padj < 0.01). Dysregulated lncRNAs (DElncRNAs) and miRNAs (DEmiRNAs) with binding sites were screened by the miRcode database (http://www.mircode.org/?gene=%20&mirfam=&class=&cons=%20&trregi%20on=). miRDB, TargetScan, and mirDIP databases were applied to predict downstream genes of miR-424-5p. Predicted results were overlapped with differentially expressed mRNAs (DEmRNAs) to acquire the targets of miR-424-5p.

### 2.2. Clinical Data and Tissue Sources

76 pairs of paired primary glioma tissue and the corresponding adjacent normal tissue were acquired. The samples were collected from patients treated with surgical resection in Xi'an International Medical Center Hospital from October 2018 to October 2019, and their disease was confirmed by experienced pathologists. Acquired tissue was quickly frozen in liquid nitrogen and then stored in an -80°C refrigerator. Informed consent was signed by patients. Clinicopathological data of patients are presented in Supplementary Table1.

### 2.3. Cell Lines and Cell Culture

Human astrocytes HEB and human glioma cell lines T98G, A172, SNB19, and U251 were provided by Chinese Academy of Sciences Cell Bank (Shanghai, China). Dulbecco's Modified Eagle Medium (DMEM) +10% fetal bovine serum (FBS) was utilized for cell cultivation. The plates were cultivated routinely. Information of cell lines was exhibited in Supplementary Table2.

### 2.4. Cell Transfection

The overexpression of miR-424-5p was gained by transfection of miR-424-5p mimic (Genepharma, Shanghai, China). FAM87A-pcDNA3.1 vector (GeneCopoecia, Guangzhou, China) was employed for the overexpression of FAM87A. PPM1H knockout was achieved using pLent-PPM1H-shRNA vector (Guangzhou, China). Lipofectamine 2000 (Invitrogen) was utilized for cell transfection. Then, cells were cultivated for 24 h or 48 h for further detection or extraction of RNA/proteins.

### 2.5. qRT-PCR

Trizol Reagent was utilized for total RNA extraction (Invitrogen, CA, USA). The miR-424-5p expression was quantified by Hairpin-it TM miRNAs qPCR kit (GenePharma, Shanghai, China) with U6 as an internal reference. SYBR Green qPCR (Takara, Dalian, China) was employed to detect FAM87A and PPM1H. 36B4 and GAPDH were utilized as internal references of FAM87A and PPM1H, respectively. Primers were listed in Supplementary Table3.

### 2.6. Western Blot

Cells were lysed with radioimmunoprecipitation assay buffer containing 1% phenylmethanesulfonyl fluoride (PMSF). Protein lysate was loaded on sodium dodecyl sulfate polyacrylamide gel. Then, proteins were transferred onto a polyvinylidene fluoride (PVDF) membrane. Later, the membrane was cultivated with primary antibodies overnight at 4°C, after which was a cultivation with secondary antibody labeled with horseradish peroxidase. At last, ECL substrates were applied to visualize protein bands (Millipore, MA, USA). The information of antibodies was offered in Supplementary Table4.

### 2.7. RNA Binding Protein Immunoprecipitation (RIP) Assay

Briefly, 100 *μ*l nuclear extract was diluted to 1 mL with nuclear lysis buffer. The samples were incubated with agarose beads with anti-AGO2 antibody or nonspecific mouse IgG overnight at 4°C (Calbiochem, San Diego, CA, USA). After samples were washed, the immunoprecipitated RNA was extracted with TRIzol Reagent (Takara Bio) and dissolved in nuclease-free water. Then, RNA was measured by qRT-PCR.

### 2.8. MTT and EdU Assays

Cells were inoculated in 96-well plates. At each specific time, cells were incubated with 100 *μ*L MTT solution and then cultured at 37°C for 3 h. After cultivation, each well was put in 150 *μ*l solvent, wrapped with aluminum foil, and shaken well for 15 min. Absorbance was then measured at 490 nm. Each assay was carried out 3 times. For the treatment group of TMZ (Sigma-Aldrich, USA), the final concentration of TMZ was 80 *μ*mol/L when TMZ was added into experimental cells. The drug in the control group was dimethyl sulfoxide (DMSO).

EdU kit (RiboBio, Guangzhou, China) was applied to measure cell DNA synthesis rate. EdU-positive cells were counted by microscopy under the 3 randomly selected fields. The ratio of EdU-positive cells (red fluorescence) to Hoechst-stained cells (blue fluorescence) was employed to evaluate cell proliferative activity.

### 2.9. Transwell Assays

Cell migratory and invasive capacities were detected through 24-well transwell chambers. In the migration assay, 1 × 10^5^ cells were inoculated with 200 *μ*L serum-free medium in the upper chamber and DMEM cell medium plus 10% FBS was placed into the lower chamber. After incubation at 37°C for 24 h, invading cells were treated with 4% paraformaldehyde and crystal violet. Next, numbers of stained cells were counted and imaged by the microscopy. In the invasion test, the upper chamber was coated with matrix (BD Bioscience, USA), and the rest steps are the same as the migration assay.

### 2.10. Dual-Luciferase Assay

Cells were cotransfected with miR-424-5p mimic and corresponding luciferase reporter vectors (FAM87A and PPM1H). Luciferase activity was examined with Luciferase Assay Reagent (Promega, Fitchburg, WI, USA) 48 h after transfection.

### 2.11. Fluorescence In Situ Hybridization (FISH) and Subcellular Isolation

The FISH assay was conducted with Ribo Fluorescent In Situ Hybridization Kit and Ribo lncRNA Fish Probe Mix (Ribo, Guangzhou, China). The separation of nucleus and cytoplasm was conducted using PARIS Kit (Life Technologies, Carlsbad, USA) in line with specifications.

### 2.12. Immunohistochemical (IHC) Analysis

Frozen glioma or mouse tumor specimens were cut into 5 *μ*m sections and placed on a glass slide covered with polylysine (Sigma-Aldrich). Then, they were air dried and fixed with acetone. IHC was carried out as described in the literature [12]. Image-Pro Plus v.6.2 software (Media Cybernetics, Rockville, MD, USA) was employed to assess positive pixel intensity as integrated optical density, with uniform settings for all slides. Percentage of the immunoreactive area of each protein in the total section area was calculated. Values were presented as mean ± standard deviation.

### 2.13. Tumor Xenotransplantation Assay

Twelve female BALB/C nude mice (5 weeks old; Vital River, Beijing, China) were kept under certain pathogen-free conditions. In vivo assays were carried out in line with the Guidelines for the Use of Experimental Animals. Specifically, a stable transduction cell line with overexpressed FAM87A and a control cell line were constructed, and then they were, respectively, inoculated into the left armpit of the mice. The mice were divided into experimental groups and control groups. Then, in line with the volume formula (1/2 × length × width^2^), the size of the tumor was measured with a vernier caliper every week. In the fourth week, all mice were sacrificed, and tumors were weighed. The removed tumor mass was utilized in subsequent experiments.

### 2.14. Data Analysis

Data analysis was performed utilizing GraphPad Prism 7. Data were listed as mean ± standard deviation from at least 3 replicates, and differences between groups were compared through unpaired two-tailed student *t*-test. Pearson correlation coefficient was applied to evaluate relationship between FAM87A and miR-424-5p. Kaplan-Meier and Cox regression analyses were employed to determine the relationship between FAM87A and overall survival and prognosis of glioma. *p* < 0.05 was thought to be statistically significant.

## 3. Results

### 3.1. FAM87A Is Lowly Expressed in Glioma Tissue and Cells and Negatively Correlated with TNM Staging and Metastasis

By edge*R* differential analysis, a total of 557 DElncRNAs and 59 DEmiRNAs were obtained (Figure 1(a)). The differences were compared in the miRcode database. Then, 35 lncRNAs and 8 miRNAs were found to have binding sites. FAM87A was one of the DElncRNAs. Survival curves expressed that overall survival time of glioma patients with restrained FAM87A was shorter than those with less expressed FAM87A (Figure 1(b)). The FAM87A expression in 76 pairs of glioma tissue and adjacent normal tissue was examined by qRT-PCR. In comparison with corresponding adjacent normal tissue, the FAM87A expression was low in glioma tissue (Figure 1(c)). Moreover, compared with glioma patients with nonmetastatic tumors, FAM87A was suppressed in patients with metastatic tumors (Figure 1(d)) and decreased markedly with the increase of pathological stage (Figure 1(e)). Combined with clinical sample information, we unveiled that FAM87A was not correlated with patients' age, sex, tumor size, tumor location, and differentiation degree. However, FAM87A was prominently correlated with lymphatic metastasis and TNM (Supplementary Table 1). Besides, we analyzed expression differences of FAM87A between low grade glioma (LGG) and glioblastoma (GBM) based on the TCGA database, whose result was consistent with the prior experiments (Figure 1(f)). Finally, qRT-PCR detection results indicated that FAM87A in human glioma cell lines was remarkably downregulated (Figure 1(g)). Among 4 glioma cell lines, FAM87A was relatively low in T98G and A172. Hence, they were selected for subsequent in vitro experiments, while T98G was used for in vivo experiments.

### 3.2. Overexpression of FAM87A Inhibits Malignant Progression of Glioma

Cell line with the FAM87A overexpression was constructed for further detection. The results of the MTT assay expressed that the FAM87A overexpression evidently reduced T98G and A172 cell viability (Figure 2(a)). The EdU assay also suggested that reproductive activity of T98G and A172 cells was notably inhibited after the overexpression of FAM87A (Figure 2(b)). The transwell assay uncovered that the number of migrating and invading cells was notably reduced after the overexpression of FAM87A (Figure 3(a)). Western blot detected the expression levels of invasion- and metastasis-related proteins, and the results also suggested that fibronection, N-cadherin, vimentin, MMP9, and MMP2 expressions declined while E-cadherin increased after the overexpression of FAM87A (Figure 3(b)). The influence of fostered FAM87A on the resistance of cells to TMZ was tested, uncovering that the resistance of both kinds of cancer cells to TMZ decreased prominently after the overexpression of FAM87A (Figure 3(c)). According to the above experimental data, FAM87A may play a part as a tumor inhibitor in malignant development of glioma. The results of FISH and subcellular isolation indicated that FAM87A was basically distributed in the cytoplasm (Figure 2(c)).

### 3.3. FAM87A Acts as a Sponge of miR-424-5p in Glioma Cells

First, downstream modulatory miRNAs of FAM87A were predicted in the miRcode database and intersected with DEmiRNAs to obtain 5 miRNAs (miR-424, miR-96, miR-195, miR-497, and miR-93) (Figure 4(a)). Only miR-424 was negatively relevant with prognosis (Figure 4(b)) and could promote the occurrence of variety types of cancers, which could be employed as a potential marker [13, 14]. Therefore, miR-424-5p was selected for further exploration. Compared with paracancerous tissue, the miR-424-5p expression in the glioma tissue was upregulated and negatively associated with the expression level of FAM87A (Figures 4(c) and 4(d)). Binding sites of FAM87A and miR-424-5p were predicted utilizing miRcode. Results of dual-luciferase reporter genes revealed that hastened miR-424-5p restrained expression of cells with wild-type (WT) FAM87A but had no effect on the expression of cells with mutant (MUT) FAM87A. A binding relationship between miR-424-5p and FAM87A was displayed (Figure 4(e)). Result was further confirmed by the RIP assay (Figure 4(f)). In addition, the influences of boosted FAM87A on miR-424-5p in T98G and A172 cells were detected. Results unveiled that the miR-424-5p expression in cells with overexpressed FAM87A was prominently decreased (Figure 4(g)). These findings presented that in glioma, miR-424-5p was directly acted by FAM87A, and FAM87A interacted with miR-424-5p to constrain activity of miR-424-5p.

Then, rescue experiments were carried out in glioma cell lines T98G and A172. According to MTT results, the cell activity was markedly increased after the overexpression of miR-424-5p while it was markedly inhibited after the overexpression of miR-424-5p and FAM87A simultaneously (Figure 5(a)). Evidently, more cancer cells migrated and invaded after fostering miR-424-5p, while these abilities were decreased after accelerating miR-424-5p and FAM87A together (Figure 5(b)). After boosting miR-424-5p, resistance of cells to TMZ increased remarkably, while resistance of cells to TMZ was weakened when miR-424-5p and FAM87A were fostered concurrently (Figure 5(c)). These results suggested that FAM87A may directly modulate the development of glioma cells via interacting with miR-424-5p.

### 3.4. FAM87A Boosts PPM1H via Inhibiting miR-424-5p

Downstream regulatory target genes of miR-424-5p were predicted by the bioinformatic database, and then the predicted results were overlapped with the DEmRNAs and 9 DEmRNAs (PPM1H, ANKRD33B, PCDHAC2, RSPO3, SPTBN2, UNC13A, KIF5A, SYT4, and HTR2A) with binding sites that were acquired (Figures 6(a) and 6(b)). There was a high correlation between FAM87A and PPM1H, and PPM1H was prominently positively associated with survival rate of patients with glioma (Figures 6(c) and 6(d)). Hence, PPM1H was selected as the study object. qRT-PCR results expressed that PPM1H was notably repressed in the glioma tissue, positively relevant with FAM87A and negatively relevant with miR-424-5p (Figure 6(e)). At cellular level, effects of FAM87A and miR-424-5p on the PPM1H protein expression were investigated. The results indicated that FAM87A hastened the expression of PPM1H, while the overexpression of miR-424-5p suppressed PPM1H (Figure 6(f)). The binding sites of miR-424-5p and PPM1H were found by Targetscan. Dual-luciferase reporter gene assay results indicated that facilitated miR-424-5p decreased the luciferase activity of cells with PPM1H 3′-UTR WT, while luciferase activity of cells with PPM1H 3′-UTR MUT was not affected (Figure 6(g)). RIP test on T98G cells showed that the overexpression of FAM87A could restrain binding of PPM1H and miR-424-5p (Figure 6(h)), indicating that FAM87A was highly likely to competitively bind to miR-424-5p with PPM1H, thereby modulating the development of glioma.

Furthermore, sh-PPM1H was used to construct cell line with si-PPM1H, and role of PPM1H in glioma was explored through a series of cell functions. The MTT assay results indicated that silencing PPM1H promoted the viability of T98G and A172 cells (Figure 6(i)). Transwell results demonstrated that migration and invasion of T98G and A172 cells were markedly enhanced after PPM1H silence (Figure 6(j)). The influence of silencing PPM1H on the resistance of cells to TMZ was tested, finding that the resistance of both cancer cells to TMZ increased remarkably after silencing PPM1H (Figure 6(k)). These results displayed that PPM1H, as a tumor suppressor in glioma, could constrain biological functions of glioma. FAM87A may modulate PPM1H to mediate the development of glioma through binding to miR-424-5p competitively.

### 3.5. PI3K/Akt Signaling Pathway Is Regulated by FAM87A/miR-424-5p/PPM1H Signaling axis

Above results proved, the FAM87A/miR-424-5p/PPM1H signaling axis regulated the biological function of glioma. Then, we further explored the potential signaling pathway. Through the Kyoto Encyclopedia of Genes and Genomes (KEGG) pathway enrichment analysis on FAM87A/miR-424-5p/PPM1H, we found that all 3 kinds of RNA were enriched in the phosphatidylinositol signaling pathway (Supplementary Figure 1). The PI3K/Akt pathway was most closely relevant to proliferation and metastasis of cancer. To dig whether the FAM87A/miR-424-5p/PPM1H signaling axis modulated the PI3K/Akt signaling pathway, we hastened FAM87A or silenced PPM1H in T98G and A172 cells to determine its influences on PI3K and Akt. The findings expressed that expression levels of p-PI3K and p-Akt in T98G and A172 cells were remarkably downregulated after overexpressing FAM87A while they were remarkably upregulated after silencing PPM1H. Expressions of p-PI3K and p-Akt were not evidently different from those of the blank group after silencing PPM1H and overexpressing FAM87A together (Figure 7(a)). As demonstrated by these results, the FAM87A/miR-424-5p/PPM1H signaling axis may modulate the PI3K/Akt signaling pathway.

### 3.6. FAM87A Inhibits Tumor Growth In Vivo

Cells with the mimic vectors were injected into the left axilla of mice as a control. Results unveiled that tumor growth was remarkably constrained in the overexpression group of FAM87A in comparison with the blank group (*p* < 0.05) (Figure 8(a)). Tumors with overexpressed FAM87A were smaller and lighter than the control tumors (Figures 8(b) and 8(c)). In addition, IHC suggested a decline in the Ki67 expression and a boosting PPM1H expression in the tumor with overexpressed FAM87A (Figures 8(d) and 8(e)). Expression levels of invasion- and metastasis-related proteins were detected after the overexpression of FAM87A. It was uncovered that the expression of fibronection, N-cadherin, vimentin, MMP9, and MMP2 were declined while E-cadherin expression was facilitated after the overexpression of FAM87A (Figure 8(f)). By these results presented, FAM87A inhibited tumor growth in vivo.

## 4. Discussion

Glioma is a malignant tumor in brain tumors, with vascular hyperplasia, strong invasion, and poor prognosis [15]. Most glioma patients are difficult to cure due to the development of resistance to traditional treatment drugs [16]. In recent years, increasing evidence showed that lncRNAs are involved in regulation of tumor progression [17]. Based on previous bioinformatic analyses, FAM87A may act as a tumor suppressor in glioma, inhibiting proliferative, migratory, and invasive capacities. In this paper, we revealed that FAM87A was downregulated in glioma tissue and cells, and it was associated with clinical characteristics. Overall survival time of glioma patients with suppressed FAM87A was shorter than that of glioma patients with high expression of FAM87A, and FAM87A was negatively relevant with TNM staging and metastasis. Further, in vivo and in vitro assays jointly manifested that overexpressing FAM87A evidently suppressed the progression of glioma cells as well as tumor growth in vivo. Above findings all proved that FAM87A constrained the malignant progression of glioma.

The interaction between lncRNAs and miRNAs is the main factor modulating the proliferation, invasion, and migration of cancer cells [18]. Yao et al. [19] presented that knockout of lncRNA XIST in glioma cells induced upregulation of miR-152, thereby inhibiting cell proliferation, invasion, and migration. Zhang et al. [20] uncovered that H19 is closely related to pathological types of glioma in different glioma tissue microarray data sets. They found that H19 regulates CDH1 by binding to miR-675, thereby affecting glioma growth and recurrence. Moreover, the H19 expression also affects the sensitivity of TMZ to chemotherapy [20]. Here, the overexpression of miR-424-5p combining boosted FAM87A could reverse the effect of overexpressing miR-424-5p alone on biological function of glioma. This suggested that, as a sponge of miR-424-5p, FAM87A modulated cell proliferative, migratory, and invasive capacities.

Microarray analysis and luciferase assay proved that miR-424-5p had binding sites with PPM1H, and miR-424-5p acted directly on PPM1H. In glioma tissue and cells, FAM87A was downregulated, miR-424-5p was facilitated, and PPM1H was repressed. There was a negative correlation between miR-424-5p and PPM1H, while a positive relationship between FAM87A and PPM1H. The biological functions of PPM1H on human cells are to control cell proliferation and differentiation [21–24]. Han Zhu et al. [25] demonstrated that PPM1H is constrained in pancreatic cancer cells, silencing PPM1H could induce epithelial-mesenchymal transition (EMT) in BXPC-3 cells and accelerated cell invasion, and metastasis, and PPM1H may function as a new tumor suppressor. In this article, PPM1H was lowly expressed in glioma tissue, and silencing PPM1H prominently boosted proliferation, migration, and invasion of cancer cells. These findings indicated that in glioma, FAM87A could restrain the development of glioma by targeting PPM1H through the sponge of miR-424-5p. In addition, investigation on the downstream pathway of the FAM87A/miR-424-5p/PPM1H signaling axis revealed that it may regulate the PI3K/Akt pathway (Figure 7(b)). Many experiments proved that the PI3K/Akt pathway is closely related to multiple biological functions of a variety of tumors^26^–^29^. Therefore, the effects of the FAM87A/miR-424-5p/PPM1H signaling axis on the biological activities of glioma cell progression and drug resistance may be partly due to the regulation of the PI3K/Akt signaling pathway.

Taken together, FAM87A as a tumor eliminator was downregulated in glioma. FAM87A could restrain progression of glioma through targeting PPM1H through sponge of miR-424-5p, while the FAM87A/miR-424-5p/PPM1H signaling axis can modulate the PI3K/Akt signaling pathway. In a word, the FAM87A/miR-424-5p/PPM1H axis plays a crucial part in glioma and can be utilized as a key treatment target.

## Figures and Tables

**Figure 1:** FAM87A is lowly expressed in glioma and negatively correlated with pathological stage and metastasis. (a) Volcano map of DElncRNAs and DEmiRNAs in glioma. (b) Kaplan-Meier analysis for FAM87A. (c) FAM87A expression in 76 pairs of glioma tissue and adjacent tissue examined by qRT-PCR. (d) FAM87A expression in 76 metastatic (N0) and nonmetastatic (NX) glioma tissues tested by qRT-PCR. (e) FAM87A expression in the stages of I, II, and III + IV in 76 glioma tissues examined by qRT-PCR. (f) FAM87A expression in LGG and GBM based on the TCGA database. (g) FAM87A expression in astrocytes (HEB) and glioma cells (T98G, A172, SNB19, and U251) detected by qRT-PCR; ^∗^*p* < 0.05 and ^∗∗^*p* < 0.01. Plus: when logFC>2 and -log10(FDR)>2, it is a differentially up-regulated gene, when logFC2, it is a differentially downregulated gene.

**Figure 2:** The overexpression of FAM87A inhibits glioma cell proliferation and localization of FAM87A in tissue and cells. (a) Growth activity of T98G and A172 cells after the FAM87A overexpression measured by the MTT assay. (b) Proliferation of T98G and A172 cells after the FAM87A overexpression measured by the EdU assay. (c) FISH was used to locate the position of FAM87A in glioma tissue; qRT-PCR detected GAPDH, U6, and FAM87A expressions after nuclear and cytoplasmic separation in T98G and A172 cells; ^∗^*p* < 0.05.

**Figure 3:** The overexpression of FAM87A inhibits migration, invasion, and TMZ drug resistance of glioma cells. (a) Migration and invasion of T98G and A172 cells after facilitated FAM87A were assessed using the transwell assay (×100). (b) The expression level of EMT-related proteins after the FAM87A overexpression was evaluated by western blot. (c) Influence of T98G and A172 cells on TMZ drug resistance after the FAM87A overexpression detected by the MTT assay; ^∗^*p* < 0.05.

**Figure 4:** FAM87A inhibits the miR-424-5p expression. (a) The Venn diagram of predicted target miRNAs and DEmiRNAs. (b) The relationship between the miR-424 expression and overall survival time of glioma patients analyzed by Kaplan-Meier. (c) MiR-424-5p is hastened in glioma. (d) Interaction between miR-424-5p and FAM87A in glioma tissue. (e) Dual-luciferase reporter gene assay was applied to determine the interaction between FAM87A and miR-424-5p. (f) The immunoprecipitation of FAM87A and miR-424-5p in T98G cells detected by the RIP assay. (g) qRT-PCR was introduced for analyzing the expression level of miR-424-5p in T98G and A172 cells after the overexpression of FAM87A; ^∗∗^*p* < 0.01.

**Figure 5:** Effects of the FAM87A/miR-424-5p signaling axis on proliferation, migration, invasion, and resistance to TMZ of glioma cells. (a) Viability of T98G and A172 cells in each treatment group evaluated by MTT. (b) Migration and invasion of T98G and A172 cells in each treatment group evaluated by transwell assay (×100). (c) The resistance of T98G and A172 cells to TMZ in each treatment group detected by MTT; ^∗^*p* < 0.05 and ^∗∗^*p* < 0.01.

**Figure 6:** FAM87A boosts the PPM1H expression by inhibiting miR-424-5p. (a) Volcano map of DEmRNAs in glioma. (b) Venn diagram of the intersection of target mRNAs of miR-424-5p and DEmRNAs predicted by the three databases (miRDB, TargetScan, and mirDIP). (c) Kaplan-Meier analysis for PPMIH. (d) Correlation analysis between miR-424-5p and the potential targets. (e) The expression of PPM1H in 76 glioma and adjacent tissues examined by qRT-PCR and correlation analysis of FAM87A and miR-424-5p. (f) PPM1H protein expression level in T98G and A172 cells after fostered FAM87A and miR-424-5p examined by western blot. (g) The binding relationship between PPM1H and miR-424-5p confirmed by dual-luciferase reporter gene assay. (h) T98G cell line used for RIP to detect the competitive binding of miR-424-5p between FAM87A and PPM1H. (i) The growth activity of T98G and A172 cells determined by MTT after PPM1H silencing. (j) Migration and invasion of T98G and A172 cells after PPM1H silencing detected by transwell (100×). (k) The influence of T98G and A172 cells on TMZ resistance after PPM1H silencing detected by MTT; ^∗^*p* < 0.05 and ^∗∗^*p* < 0.01.

**Figure 7:** PI3K and Akt expressions in glioma cells is regulated by FAM87A and PPM1H. (a) Expression of p-PI3K, total PI3K (PI3K), p-Akt, and total Akt (Akt) protein in T98G and A172 cells. (b) Schematic diagram of regulation of tumor characteristics by FAM87A/miR-424-5p/PPM1H axis in glioma, blue lines represent downregulation.

**Figure 8:** FAM87A inhibits tumor growth in vivo. (a) Tumor growth curves of glioma in nude mice after boosted FAM87A and blank treatment, the value is presented as mean ± standard deviation (*n* = 6/group). (b) The overexpression of FAM87A inhibits tumor growth of glioma in nude mice. (c) Tumor weight of the blank group and overexpressed FAM87A group. (d) PPM1H and Ki67 expressions in tumor tissue of nude mice examined by IHC. (e) The histogram of relative expression level of PPM1H and Ki67. (f) The expression of EMT-related proteins in tumor tissue after the overexpression of FAM87A detected by western blot; ^∗^*p* < 0.05 and ^∗∗^*p* < 0.01.

## Data Availability

The data used to support the findings of this study are included within the article. The data and materials in the current study are available from the corresponding author on reasonable request.

## Supplementary Materials

Supplementary 1 Supplementary Figure 1: pathway enrichment analysis of FAM87A, miR-424, and PPM1H. (a) GSEA result of FAM87A. (b) GSEA result of miR-424. (c) GSEA result of PPM1H.

Supplementary 2 Supplementary Table 1: correlation analysis of FAM87A expression and pathological parameters in glioma tissue.

Supplementary 3 Supplementary Table 2: cell lines utilized in this study.

Supplementary 4 Supplementary Table 3: primer sequences utilized in the study.

Supplementary 5 Supplementary Table 4: antibodies utilized in the study.
